This article has been retracted.

# Resistance to DDT and Pyrethroids and Increased kdr Mutation Frequency in *An. gambiae* after the Implementation of Permethrin-Treated Nets in Senegal

**DOI:** 10.1371/journal.pone.0031943

**Published:** 2012-02-22

**Authors:** Mamadou O. Ndiath, Seynabou Sougoufara, Abdoulaye Gaye, Catherine Mazenot, Lassana Konate, Oumar Faye, Cheikh Sokhna, Jean-Francois Trape

**Affiliations:** 1 Institut de Recherche pour le Développement, Unité de Recherche sur les Maladies Infectieuses et Tropicales Emergentes (URMITE) UMR 198, Campus commun UCAD-IRD de Hann, BP 1386, CP 18524, Dakar, Sénégal; 2 Laboratoire Ecologie Vectorielle et Parasitaire, UCAD, Fann Dakar, Sénégal; Institut Pasteur, France

## Abstract

**Introduction:**

The aim of this study was to evaluate the susceptibility to insecticides of *An. gambiae* mosquitoes sampled in Dielmo (Senegal), in 2010, 2 years after the implementation of Long Lasting Insecticide-treated Nets (LLINs) and to report the evolution of kdr mutation frequency from 2006 to 2010.

**Methods:**

WHO bioassay susceptibility tests to 6 insecticides were performed on adults F0, issuing from immature stages of *An. gambiae* s.l., sampled in August 2010. Species and molecular forms as well as the presence of L1014F and L1014S kdr mutations were assessed by PCR. Longitudinal study of kdr mutations was performed on adult mosquitoes sampled monthly by night landing catches from 2006 to 2010.

**Findings:**

No specimen studied presented the L1014S mutation. During the longitudinal study, L1014F allelic frequency rose from 2.4% in year before the implementation of LLINs to 4.6% 0–12 months after and 18.7% 13–30 months after. In 2010, *An. gambiae* were resistant to DDT, Lambda-cyhalothrin, Deltamethrin and Permethrin (mortality rates ranging from 46 to 63%) but highly susceptible to Fenitrothion and Bendiocarb (100% mortality). There was significantly more RR genotype among *An. gambiae* surviving exposure to DDT or Pyrethroids. *An. arabiensis* represented 3.7% of the sampled mosquitoes (11/300) with no kdr resistance allele detected. *An. gambiae* molecular form M represented 29.7% of the mosquitoes with, among them, kdr genotypes SR (18%) and SS (82%). *An. gambiae* molecular form S represented 66% of the population with, among them, kdr genotype SS (33.3%), SR (55.6%) and RR (11.1%). Only 2 MS hybrid mosquitoes were sampled and presented SS kdr genotype.

**Conclusion:**

Biological evidence of resistance to DDT and pyrethroids was detected among *An. gambiae* mosquitoes in Dielmo (Senegal) within 24 months of community use of LLINs. Molecular identification of L1014F mutation indicated that target site resistance increased after the implementation of LLINs.

## Introduction

Recently, huge progress has been made in the control of malaria in Sub Saharan African countries [1], [2]. In Senegal, between 2006 and 2009, malaria proportional morbidity fell from 33.57% to 3.1%. During the same period, proportional mortality decreased from 18.17% to 4.4% [3]. These changes followed the introduction of new prevention, diagnostic and treatment polices [4]. As recommended by WHO, control strategy included actions to targeting malaria parasite vectors including indoor residual spraying (IRS), the use of long-lasting insecticide-treated bed nets (LLINs) and the destruction of larvae breeding sites [5]. The major challenge faced by vector control programs is the development of resistance to insecticides [6]. In recent years, the widespread use of insecticides in agriculture [7] but also for bed net treatment [8], [9] contributed to the selection of resistant mosquito strains. Resistance to pyrethroids is a particular threat for malaria control, since they are currently the only recommended and approved insecticides for treating bed nets, primarily because of their low toxicity for humans compared to other pesticides [10].

Mosquitoes' resistance to insecticide has been demonstrated by both *in vivo* biological test and by the identification of resistance alleles in a vast number of sites across Africa. Especially, kdr mutation genotype has been recognized to be related to DDT and pyrethroid resistance [11]. *An. gambiae s.l.* and *An. funestus* are the two major malaria vectors in Dielmo (Senegal) [12]; both have previously been found to be potentially resistant to pyrethroids [13], [14]. The resistance to insecticide has been shown to be locally highly variable even inside a country or a region [15]–[19]. An early detection of resistance is necessary for the implementation of rational vector control programs [20]. It will not be possible to have reliable information without a regular and tight mapping of the resistance status of mosquitoes.

Since 1990, an epidemiological study is ongoing in Dielmo (Senegal) that involves long-term investigations on host-parasite relationships and mechanisms of protective immunity in residents of this Senegalese village [21]. For the first time in Senegal, universal coverage with LLINs (Permanet® 2.0) was implemented in Dielmo in July 2008. After a dramatic decrease in malaria morbidity observed after the implementation of LLINs, a rebound was observed in this village 2 years later [22]. In order to identify the causes for increased morbidity, a study of mosquito susceptibility to insecticide was needed. This paper reports the evolution of the presence of kdr mutation, in *Anopheles gambiae s.l.*, 2 years before and after the implementation of LLINs and the results of resistance tests to 6 frequently used insecticides performed in 2010, 2 years after the implementation of LLINs.

## Methods

### Mosquito sampling

This study is part of the Dielmo Project that has been described in detail elsewhere [21]. Briefly, the village of Dielmo (13°43N, 16°24W) is located 280 km Southeast of Dakar and about 15 km north of the Gambian border in an area of Sudan-type savannah. About 400 inhabitants are living in the village. Rainfall occurs during a four-month period, from June to October. Dielmo is situated on the marshy bank of a small permanent stream, with anopheles larval sites present all year round.

Adult mosquitoes were collected by human landing catches (HLC) monthly from July 2006 to December 2010. Night captures (7:00 PM–7:00 AM) were conducted once or more times each month in two indoor and two outdoor sites. In each site, two trained collectors (adult male volunteers) worked alternatively for one hour and rested for one hour. Anopheline identification was performed following the Gillies and DeMeillon morphologic identification keys [23]. Mosquitoes belonging to the *Anopheles gambiae sensus lato (s.l.)* group were stored for following steps.

In August 2010, during the rainy season, immature stages of *An. gambiae* s.l. were collected from 10 breeding sites situated in and around the village (river, rain pools and cattle watering places). Larvae were pooled and fed with Tetramin® baby fish food locally until emergence. Unfed 2–3 days female *An. gambiae s.l.* mosquitoes were used for insecticide susceptibility tests.

### Susceptibility test

Bioassays were carried out using WHO test kits for adults mosquitoes [24] with six insecticides of technical grade quality: one belonging to the Carbamate group (0.1% Bendiocarb), one Organophosphate (1% Fenitrothion), 3 pyrethroids (0,05% Lambda-cyhalothrin, 0.05% Deltamethrin, 0,75% Permethrin) and one Organochlorine (4% DDT). Impregnated papers were obtained from the WHO reference center (Vector Control Research Unit, University Sains Malaysia, Penang, Malaysia). Tests were performed with batches of 25 *An. gambiae s.l*., with four batches tested against each insecticide. Mosquitoes were exposed to insecticide-impregnated filter paper for 1 hour at 25–27°C and 80% relative humidity. The number of knockdown mosquitoes was recorded at 10, 15, 20, 30, 40, 50, 60 and 80 min. After exposure, mosquitoes were kept in observation tubes and supplied with a 10% sugar solution. Mortality was recorded after 24 hours. The mortality of a control stain of *An. gambiae* (Yaoundé known to be 100% susceptible to all tested insecticides [25], [26]) was studied as a positive control. Batches exposed to untreated papers were used as negative control. Since mortality in negative controls was always <5%, no adjustment was performed for treated batches. For each insecticide, a sample of 50 *An. gambiae s.l.* specimens was randomly selected, including equal numbers of dead and surviving specimens (when available) and used for molecular tests.

### Molecular identification and kdr genotyping

In the subsample of mosquitoes used for bioassay and in adults sampled by HLC during the longitudinal study, detection of L1014F and L1014S kdr mutations (thereafter identified as kdr-w and kdr-e respectively) was performed by PCR [27], [28]. Mosquitoes used for bioassay were identified down to their species and molecular form with the PCR RFLP method [29].

### Data analysis

WHO (1998) criteria were used to evaluate the resistance/susceptibility status of the tested mosquito populations (<80% mortality: resistance, 80–98% mortality: increased tolerance, >98% mortality: susceptibility) [24]. Fifty and 95 percent knockdown times (respectively KDT_50_ and KDT_95_) were computed with probit regression models. Rates were compared using Fisher exact and Pearson Chi^2^ tests. Statistical analyses were performed using Stata 10.1 software. A P value of 0.05 or less was considered as significant.

### Ethics approval

The Dielmo project was initially approved by the Ministry of Health of Senegal and the assembled village population. Approval was then renewed on a yearly basis. Audits were regularly conducted by the National Ethics Committee of Senegal and ad-hoc committees of the Ministry of Health, the Pasteur Institute and the Institut de Recherche pour le Développement.

## Results

### Kdr genotype dynamic in adult *An. gambiae s.l.*

From July 2006 to December 2010, no specimen with L1014S (kdr-e) mutation was identified.

The repartition of kdr genotype during the study period is presented in Figure 1. Before the implementation of LLINs, L1014F allelic frequency was low and not different when comparing 24-13 months and 12-0 months before periods (2.0 and 3.5% respectively, Chi^2^ = 1.4, p = 0.24). This rate significantly increased to 4.6% within the first 12 months that followed the distribution of LLINs (Chi^2^ = 4.4, p<0.05 vs. pre-implementation) and again 13–30 months after to 18.7% (Chi^2^ = 70, p<0.001 vs. preceding period) (Figure 1).

**Figure 1:** kdr mutation in *An. gambiae* before and after the implementation of LLINs. Proportion (and 95% CI) of *An. gambiae* with L1014F homozygote mutation (RR), heterozygote mutation (RS) or wild type (SS) sampled 24-13 months (n = 228) and 12-0 months (n = 99) before the implementation of long lasting insecticide-treated nets (LLINs) in July 2008, 0–12 months (n = 327) and 13–30 months after (n = 582).

### Sensitivity to insecticides in 2010

Mortality data indicated that mosquitoes were highly resistant to 4 of the 6 insecticides tested including DDT and all Pyrethroids (Deltamethrin, Lambda-cyhalothrin and Permethrin). Mortality rates ranged from 46 to 63%, far below the susceptibility limit of 80% (Table 1). Mosquitoes were totally susceptible to Fenitrothion (Organophosphate) and Bendiocarb (Carbamate) with a 100% mortality observed for both insecticides.

**Table 1:** Bioassay susceptibility tests in 2010.

	Mortality %	95% CI	KDT_50_	95% CI	KDT_95_	95% CI
**Deltamethrin 0,05%**	63	[53.5–72.5]	28.0	[25.3–30.7]	na	-
**Lambda-cyhalothrin**	60	[50.3–69.7]	43.6	[40.9–46.3]	na	-
**Permethrin 0,75%**	46	[36.2–55.8]	48.7	[45.5–51.9]	na	-
**DDT 4%**	61	[51.4–70.6]	64.6	[58.1–71.0]	na	-
**Fenitrothion**	100	-	70.4	[67.1–73.7]	na	-
**Bendiocarb 0,1%**	100	-	17.5	[16.4–18.5]	39.0	[37.9–40.0]

Mortality rate (%) 24 hours after exposition, 50 and 95% knockdown (KDT_50_ KDT_95_) time (min) with 95% confidence interval (CI), obtained on 100 *An. gambiae* for each insecticide tested. na: not applicable, 95% knock down time exceeded 80 min.

Knockdown time 50 (KDT_50_) was higher than 40 minutes for Lambda-cyhalothrin, Permethrin, DDT and Fentrothion and KDT_95_ exceeded the 80-min observation period (Table 1). Knockdown time was shorter for Deltamethrin (KDT_50_ = 28.0 min) and even shorter for Bendiocarb (KDT_50_ = 17.5 and KDT_95_ = 39.0 min).

In the 300-specimens sample selected for molecular analysis among dead and surviving mosquitoes, 11 (3.7%) were *An. arabiensis*, 89 (29.7%) *An. gambiae s.s.* molecular form M, 2 (0.7%) MS hybrids and 198 (66.0%) form S. When comparing the species and molecular forms of *An. gambiae s.l.* among dead and surviving mosquitoes, no association could be identified for Deltamethrin, Lambda-cyhalothrin, Permethrin and DDT (Fisher exact test p>0.2, Table 2). This analysis could not be performed for Fenitrothion and Bendiocarb since all mosquitoes died.

**Table 2:** Molecular forms of *An. gambiae s.l.* among dead and surviving mosquitoes after insecticide exposure.

		Molecular form of *An. gambiae s.l.*				Fisher exact test p
		*An. arabiensis*	M	MS	S	
**Deltamethrin 0,05%**	Dead n = 25	4% (1)	36%(9)	0%(0)	60%(15)	0.551
	Survivors n = 25	0%(0)	28%(7)	0%(0)	72%(18)	
**Lambda-cyhalothrin**	Dead n = 25	4%(1)	12%(3)	0%(0)	84%(21)	0.289
	Survivors n = 25	0%(0)	28%(7)	0%(0)	72%(18)	
**Permethrin 0,75%**	Dead n = 25	0%(0)	20%(5)	0%(0)	80%(20)	0.702
	Survivors n = 25	0%(0)	12%(3)	0%(0)	88%(22)	
**DDT 4%**	Dead n = 25	12%(3)	44%(11)	0%(0)	44%(11)	0.385
	Survivors n = 25	4%(1)	32%(8)	4%(1)	60%(15)	
**Fenitrothion**	Dead n = 50	4%(2)	42%(21)	2%(1)	52%(26)	-
**Bendiocarb 0,1%**	Dead n = 50	6%(3)	30%(15)	0%(0)	64%(32)	-
**Total**	n = 300	3.7% (11)	29.7% (89)	0.7% (2)	66.0% (198)	

Proportion and number of mosquitoes belonging to *An. arabiensis* specie and *An. gambiae s.s*. molecular form M, MS and S assessed after insecticide sensitivity in both dead and surviving (when available) mosquitoes.

### Kdr mutations and resistance phenotype

Among the 300 surviving and dead specimens selected for kdr-w identification, 152 (50.7%) were SS, 126 (42%) SR and 22 (7.3%) RR kdr-w genotype (Table 3). No specimen presented the kdr-e mutation. There was a significant difference in kdr-w genotype between dead and surviving mosquitoes for DDT and all Pyrethroids (Fisher exact p ranging from 0.041 to 0.002). R allelic frequency was significantly higher in survivors for each insecticide (Fisher exact p≤0.001). No RR genotype was identified among dead mosquitoes after DDT or pyrethroids exposure (Table 3). Among survivors, 70% of specimens presented a mutated allele; 30% had a resistant phenotype although they did not present kdr mutation.

**Table 3:** kdr-w mutation genotypes and allelic frequencies among dead and surviving mosquitoes after insecticide exposure.

		Genotype			Fisher exact test p	Allelic frequency		Fisher exact test p
		SS	SR	RR		S	R	
**Deltamethrin 0,05%**	Dead n = 25	64% (16)	36%(9)	0% (0)	0.002	82% (41)	18% (9)	<0.001
	Survivors n = 25	28% (7)	40% (10)	32% (8)		48% (24)	52% (26)	
**Lambda-cyhalothrin**	Dead n = 25	60% (15)	40% (10)	0% (0)	0.013	80% (40)	20% (10)	0.001
	Survivors n = 25	24% (6)	68% (17)	8% (2)		58% (29)	42% (21)	
**Permethrin 0,75%**	Dead n = 25	52% (13)	48% (12)	0% (0)	0.002	76% (38)	24% (12)	<0.001
	Survivors n = 25	20% (5)	52% (13)	28% (7)		46% (23)	54% (27)	
**DDT 4%**	Dead n = 25	76% (19)	24% (6)	0% (0)	0.041	88% (44)	12% (6)	<0.001
	Survivors n = 25	48% (12)	36% (9)	16% (4)		66% (33)	34% (17)	
**Fenitrothion**	Dead n = 50	50% (25)	50% (25)	0	-	75% (75)	25% (25)	-
**Bendiocarb 0,1%**	Dead n = 50	68% (34)	30% (15)	2% (1)	-	82% (83)	17% (17)	-
**Total**	n = 300	50.7% (152)	42% (126)	7.3% (22)	-	71.7% (430)	28.3% (170)	-

Proportion and number of mosquitoes with kdr-w genotype SS (sensitive, sensitive), SR (resistant, sensitive) and RR (resistant, resistant) and corresponding allelic frequency assessed after insecticide sensibility in both dead and surviving (when available) mosquitoes.

The frequency of kdr-w mutation was significantly different according to the molecular form of *An. gambiae* (Fisher exact test p<0.001, Table 4). Molecular form S had a specific kdr-w genotype compared to *An. arabiensis* and *An. gambiae s.s.* M form (Fisher exact test p<0.001 in both cases). Allelic form R was totally absent in *An. arabiensis* and in *An. gambiae* MS form. In *An. gambiae* M form, SR genotype was present (18%) and RR genotype was absent. Allele R frequency was 38.9% for molecular form S vs. 7.8% in the other groups (Fisher exact test p<0.001).

**Table 4:** kdr-w genotypes and allelic frequencies among the different molecular forms of *An. gambiae s.l*.

		Molecular form of *An. gambiae*			
		*An. arabiensis*	M	MS	S
**Kdr-w mutation**	**SS**	100% (11)	82.0% (73)	100% (2)	33.3% (66)
	**SR**	0% (0)	18.0% (16)	0% (0)	55.6% (110)
	**RR**	0% (0)	0% (0)	0% (0)	11.1% (22)
**Allelic frequency**	**S**	100% (22)	91.0% (162)	100% (4)	61.1% (242)
	**R**	0% (0)	9.0% (16)	0% (0)	38.9% (154)

Proportion and number of mosquitoes belonging to *An. arabiensis* species and *An. gambiae s.s*. molecular form M, MS and S and presenting kdr-w mutation genotypes SS, SR, and RR (Fisher exact test p<0.001) and corresponding allelic frequency.

## Discussion

The results of this study demonstrated that field population of *An. gambiae s.l.* display a high biological level of resistance to DDT and pyrethroids (Deltamethrin, Lambda-cyhalothrin and Permethrin). Similar resistance has been observed all around Africa but little information was previously published about Senegal. Investigations on the biological susceptibility to DDT performed in sentinel sites of Senegal reported a resistance to DDT in 4/10 sites [26] in 2008 and in 11/15 sites in 2010 [25]. In Africa, the resistance to DDT is widespread [15]–[18], [30] with mortality rate as low as 0% in RDC [31]. On the other hand, total susceptibility to DDT was observed in other countries [19], [32] or even in other regions of the same countries [30]. In regions where mosquitoes are still relatively susceptible to DDT, KDT_50_ is short (6–26 min) [19], whereas in regions where specimens are highly resistant to DDT, KDT_50_ is longer (more than the 80-min observation period) [18]. In our study, although resistance was detected, according to the WHO criteria, mortality rates as well as KDT_50_ were at an intermediate level.

While the resistance to pyrethroids was limited in 2008 in Senegal (detected in 0/10 sentinel sites for Deltamethrin, 2/11 for Lambda-cyhalothrin and 4/10 for Permethrin [26]), it was found to be widespread in 2010 (detected in 9/15 sites for Deltamethrin, 10/15 for Lambda-cyhalothrin and 12/15 for Permethrin [25]). Resistance to pyrethroids has been reported in various African countries [16]–[18], [30], [33]. Whilst full susceptibility to pyrethroids is still reported in other countries [19] or even in other areas of the same countries [18], [30], [34]. KDT_50_ was 49 min in our study, slightly longer than that observed in Dakar in 1995 when susceptibility was higher (77% mortality vs. 46% in our study) [14]. In studies where various pyrethroids were tested, cross-resistance or increased tolerance to all pyrethroids was confirmed [16], [17]. In our study, a cross-resistance to all pyrethroids tested was observed with low mortality rates.

In this study, the presence of kdr-w mutation was detected in *An. gambiae s.s.*; kdr-e mutation was not identified in any tested taxa. The presence of kdr mutations have been studied all around Africa [33]. While, kdr-w mutation that was initially described in Cote d'Ivoire, has been detected as far East as Uganda, kdr-e that originated in Kenya have spread into Central Africa (for review see [33]) and have recently been found in Benin [35]. Until now, kdr-e mutation has never been detected in Senegal. On the other hand, kdr-w mutation has already been observed in 2005–2006 in Senegal at a rate of 9–12% in Dakar [36] and 19% in Kedougou (Western Senegal) [37] that was lower than that observed in our study (28%). In recent studies, the allelic R frequency was found to be higher in Ghana [17], similar in RDC [31] and lower in Guinea Conakry [15]. In this study, the presence of kdr-w mutation has been shown to precede the implementation of LLINs but their rate significantly increased after.

Resistance to pyrethroids and DDT in *An. gambiae* is known to associate closely with kdr-w [11], [14], [27]. In our study, the frequency of the kdr-w allele was significantly higher in resistant-selected samples confirming the association between kdr-w mutation and the resistance phenotype to DDT and all pyrethroids tested. Moreover, a similar level of resistance was observed with DDT and all pyrethroids. Therefore a mutation of the sodium channel, that is the common target of both DDT and Pyrethroids, is likely to be involved in the observed resistance. However, 30% of specimens found among survivors presented the wild homozygote genotype. These findings support the hypothesis that target mutation is only one of the mechanisms implicated in insecticide resistance [11] and that metabolic resistance likely occurs in the *An. gambiae* population of Dielmo.

In our study, the presence of kdr-w mutation was mainly found in S molecular form of *An. gambiae*. It was absent in *An. arabiensis* and in the small sample of MS hybrids (4 specimens). Interestingly, kdr-w mutation was identified at a low rate (9%) in the M molecular form. Many studies reported the high frequency of kdr-w mutation in molecular form S in Western and Central Africa and its low frequency or absence in molecular S form (see [37] for review or recent studies [17], [31]). The kdr-w mutation, in molecular form S, has therefore spread or occurred west of the 5°W limit identified by Santolamazza *et al.* [37]. It has been hypothesized that the difference in kdr-w mutation frequency in both molecular forms was related to a different origin of the mutation in the two populations or linked to different ecological or behavioral characters between M and S forms [37].

The use of pyrethroids as pesticides for agriculture and for net treatment have both been recognized as factors responsible for the selection of resistant mosquitoes in Sub-Saharan Africa [7]–[9]. Near Dielmo, although some gardening and rice culture are performed, the use of pesticide is limited. Therefore, agriculture probably had a limited role in the emergence of the resistance to insecticides in this area. In Kenya, a lower susceptibility of *An. gambiae* to Permethrin was found in villages where Permethrin impregnated nets were implemented for one year as compared to villages without nets. The mechanism involved was postulated to include kdr mutation together with metabolic resistance [38]. In another study, an increased frequency of kdr was observed in villages with nets [39]. Insecticide treated nets were implemented in Dielmo in July 2008 as a part of the vector control study. We speculate that this may have contributed to the selection of pyrethroids resistant strains of *An. gambiae*.

In Dielmo, mosquitoes have been found to be totally susceptible to Bendiocarb, an insecticide belonging to the Carbamate class and to Fenitrothion (Organophosphate class) since we observed 100% mortality. Susceptibility of *An. gambiae* s.l. populations to Fenithrothion was also observed in all the sentinel sites in Senegal in 2008 [26] and 2010 [25]. On the other hand, a resistance to Bendiocarb appeared between 2008 and 2010 in 2/15 sentinel sites [25], [26]. In other areas, *An. gambiae s.l.* presented a resistance [15]–[17] or an increased tolerance [31] to Carbamates and increased tolerance to Malathion, another member of the Oraganophosphate class [15], [17]. In addition to pyrethroids, Carbamates (Bendiocarb and Propoxur) or Organophosphates (Fenitrothion, Malathion and Pirimiphos-methyl) are recommended by the WHO for IRS [40]. Until now, no IRS has been performed in Dielmo as part of the vector control strategy. Since complete susceptibility to Carbamates and Organophosphates has been detected in Dielmo, these insecticides should be used in priority if IRS were to be performed in this area. The reduced effectiveness of insecticides coincides with an important international effort to increase bed net coverage in African Countries in order to control malaria transmission. Notably, in Senegal 6 millions insecticide-treated nets were freely distributed to the populations between 2005 and 2010 [41], [42]. Resistance to pyrethroids is worrying, since it is the only class of insecticide safe enough to be recommended for treatment of bed nets. It appears to have a significant impact on net or IRS efficacy [43]. In Dielmo, we have recently demonstrated a rebound and age shift in malaria cases two years after the implementation of nets [22]. Since resistance of mosquitoes to several insecticides is reported in various sentinel sites in Senegal, planning alternative strategies for vector control should begin. Indeed, in Senegal, the insecticide vector resistance management started in 2011 by shifting from Deltamethrin to Bendiocarb for IRS in six selected districts. This study underlines the need to carefully document resistance and its impact on the efficacy of interventions.

In conclusion, this study demonstrated an increased frequency of kdr mutation in *An. gambiae* after the implementation of LLINs in Dielmo (Senegal). This coincided with a cross-resistance to DDT and all pyrethroids observed in 2010. Resistance was associated with a higher kdr-w allele frequency in surviving specimens. Moreover, kdr-w mutation was detected in both M and S molecular forms of *An. gambiae* and significantly more frequently in molecular form S. On the other hand, mosquitoes were fully sensitive to Bendiocarb and Fenitrothion.
